This article has been retracted.

# Continuing Care Bundle in Elderly Patients with Rectal Cancer after Radical Resection with Permanent Stoma

**DOI:** 10.1155/2022/4065886

**Published:** 2022-08-08

**Authors:** Pan Pan, Lei Chen, Dan Zhang, Shuang Rao, Ying Tao, Lin Fan

**Affiliations:** Department of Gastrointestinal Surgery, Hubei Cancer Hospital, Wuhan, Hubei, China

## Abstract

**Objective:**

A continuing care bundle can achieve a better outcome than a single implementation after discharge. This study aims to investigate the effect of this intervention in elderly patients with rectal cancer after radical resection with a permanent stoma.

**Methods:**

Elderly patients diagnosed with rectal cancer underwent radical resection with permanent stoma, they were divided into the control group (*n* = 42) and bundle group (*n* = 42). The control group received the conventional care, and the bundle group received the continuing care bundle in addition to the conventional care. At 1- and 3-month after discharge, self-efficacy, self-care knowledge, ability to change stoma appliances, negative emotions, quality of life, and patient satisfaction were observed.

**Results:**

The increased levels of self-efficacy, self-care knowledge, and ability to change stoma appliances were displayed in the bundle group after discharge as compared with that in the control group, along with the enhanced score of SF-36 subscales, including physical function (PF), role physical (RP), global health (GH) and vitality (V), social function (SF), and mental health (MH). Furthermore, patients showed alleviated depression and anxiety after the continuing care bundle as compared to those after conventional care. Besides, the bundle groups had higher patient satisfaction than the control group.

**Conclusions:**

Continuing care bundle can serve as an effectiveness intervention in elderly rectal cancer patients after radical resection with permanent stoma via increasing self-efficacy and self-care knowledge, enhancing the ability to change stoma appliance, reliving the negative emotion, and improving quality of life and patient satisfaction.

## 1. Introduction

Rectal cancer, as the 7^th^ most common cancer according to the International Agency for Research on Cancer (IARC/WHO), caused approximately 339,022 deaths with a crude rate of 4.3% in 2020 (worldwide, both sexes, all ages) [1, 2]. Similar to other malignancies, the incidence rate of rectal cancer increased with the onset of old age, and it was reported that approximately 65% patients with rectal cancer aged 65 years and older had the disease [3]. Besides, the number of elderly patients with rectal cancer who underwent surgical treatment has gradually increased along with the aging society [4]. However, 1.6%∼20.5% of patients developed anastomotic leakage following rectal cancer surgery [5], and a temporary or permanent stoma, in some cases, was necessary for treating rectal cancer in elderly patients to decrease the clinical level of anastomotic leakage as reported by several studies [6, 7]. Recent research has shown that the quality of life is perceived as worse in patients with a permanent stoma than in those without a permanent stoma [8, 9]. In addition, the stoma-related complications could cause adverse emotions and affect patients' nutritional status, thus worsening patients' long-term outcomes and quality of life [10, 11].

Even though patients are informed about guidelines and lifestyles after hospital discharge, some key ways, such as prompt medication reconciliation, medication safety, disease management, patient education, and patient-provider communication, can improve the patient's care transition, finally being associated with reduced rates of readmission, emergency department visits, and death [12, 13]. Therefore, promoting continuity of nurse care is necessary after discharge, mainly focusing on the needs and resources of the patients via taking advantage of active participation in self-care [14, 15]. A care bundle is a set of interventions, which when used together, can achieve a better outcome than a single implementation [16], thus significantly improving patient outcomes [17]. Su et al. found nurses can help rectal cancer patients with temporary stoma improve their health outcomes in stoma-specific nursing by using the evidence-based continuing care bundle via evaluating self-efficacy, the outcomes of stoma reversal, and the incidence of complications [18].

In this study, we aimed to assess the effect of a continuing care bundle on elderly rectal cancer patients after radical resection with permanent stoma, and the results showed it could increase their self-efficacy and self-care knowledge, enhance the ability to change stoma appliances, alleviate negative emotions, and improve quality of life and patient satisfaction.

## 2. Methods and Materials

### 2.1. Overall Characteristics of Patients

A total of 84 elderly patients with an average age of 77.05 ± 7.2 years (range 65∼89 years) who were diagnosed with rectal cancer by imaging and fiberoptic colonoscopy and pathological tissue test before operation were recruited between January 2019 and December 2021. Inclusion criteria: (1) patients were diagnosed as primary rectal cancer with the age >65 years; (2) patients underwent low anterior rectal resection with permanent stoma; (3) barthel index for the assessment of the activities of daily living (ADL) was more than 75 points [19]. Exclusion criteria: (1) patients had mental illness, consciousness disorder or communication disorder; (2) patients had other life-threatening diseases, such as organ failure, serious cardiovascular disease; (3) patients had abused alcohol or drugs; (4) Patients had no tumor recurrence or metastasis; (5) patients had disorder of communication, comprehension or reading; Of the 84 patients, 42 participants in the control group received the conventional care according to the previous studies, including health instruction at discharge, notice of regular follow-up visits to the hospital, and routine telephone follow-up [18, 20, 21]. Besides, the subjects in the bundle group (*n* = 42) received the continuing care bundle in addition to the conventional care.

### 2.2. Continuing Care Bundle

The patients in the bundle group received the continuing care bundle after searching the previous research as follows: (1) A team of continuing care bundle, including pharmacists, doctors, and nurses, was dispatched to evaluate the disease status in patients, including describing the current situation of stoma usage, adequate positioning of stoma. (2) After hospital discharge, once-a-week telephone follow-ups (10 to 20 minutes for each call) lasted for 3 months [22], mainly focusing on the patients' responses and questions, which were recorded and resolved on time; (3) a public WeChat account, an effective and feasible strategy to promote health education [23] was constructed to deliver the effective measures of continuing care bundles, and a WeChat group was started to fully understand the patient's condition and to correct the deficiencies during home care nursing by family members twice a week [24]. (4) Home-visiting was completed once a month for 30 mins [25] to observe the problems related to stoma and the physical recovery of patients, to deliver ostomy management reinforcement education, and to provide free medical supplies, such as ostomy bags; (5) the follow-up in an outpatient clinic mainly included the determination, solution, and self-treatment of stoma-related complications, which was written in the self-management manual [26]. At discharge, the scales listed below were fulfilled by all patients, which were then sent and collected by e-mail 1 and 3 months after discharge at the same time using the same guidance.

### 2.3. Assessment of Self-Efficacy and Self-Care Knowledge of Patients

The stoma self-efficacy scale (SSES) was adopted to test self-efficacy, which is a validated 28-item instrument with a total score of 28∼140 (higher scores indicate higher stoma-related self-efficacy) [18]. According to a previous study [27], the self-care knowledge was evaluated based on 30 items (caution in daily life: 15 items; post-surgery physical management: 6 items; the definition and status of ostomy: 2 items; aid selection and change methods: 5 items; 1 item on emotional and psychological management; and 1 item on the structure and function of the digestive organs). By judging the right/wrong answers, the total score ranged from 0–30 points.

### 2.4. Measurement for the Ability to Change Stoma Appliance

Moreover, the ability to change stoma appliances was assessed via a 4‐point scale with the total score ranging from 10 to 40 points. The higher total score indicated higher levels of self‐care knowledge and the ability to change stoma appliances.

### 2.5. Assessment for the Health-Related Quality of Life (HRQoL)

The HRQoL of patients in the two groups at hospital discharge, 3 months after discharge, and 6 months after discharge was determined using the 36-Item Short Form Health Survey questionnaire (SF-36) [28], including physical function (PF), role physical (RP), bodily pain (BP), global health (GH), vitality (V), social function (SF), role emotional (RE), and mental health (MH), with each score ranging between 0 and 100 [29].

### 2.6. Screening for Anxiety and Depression of Patients

Zung's Self-Rating Depression Scale (SDS) and Self Rating Anxiety Scale (SAS) [30], two widely-used self-report measures, were used to evaluate the depression and anxiety of patients with a total score of 100 points [31].

### 2.7. Likert 5-Point Scale

The Likert 5-Point Scale [32] was used to assess the patients' satisfaction according to a score ranging from 1 to 5, which refers to completely dissatisfied, dissatisfied, partially satisfied, satisfied, and completely satisfied, respectively.

### 2.8. Data Analysis

All data analysis were performed in GraphPad prism using *P* < 0.05 as statistical difference. The comparison of measurement data (mean ± SD) and counting data (*n*) was done using *t*-test, one-way ANOVA analysis followed by Tukey's test, Fisher's test, or *χ*^2^ test.

## 3. Result

### 3.1. Clinical and Demographic Data

There were no statistically significant differences in clinical and demographic data between the patients in the bundle group and control group at discharge (Table 1), including age (*P*=0.194), body mass index (BMI) (*P*=0.360), gender (*P*=0.814), educational level (*P*=0.826), medical payment method (*P*=0.647), living status (*P*=0.738), area of residence (*P*=0.652), smoking status (*P*=0.526), tumor/node/metastasis (TNM) stage (*P*=0.548), grade differentiation (*P*=0.541), as well as preoperative (*P*=0.823) and postoperative chemoradiotherapy (*P*=0.501).

### 3.2. The Effects of the Continuing Care Bundle on the Self-Efficacy, Self-Care Knowledge, and the Ability to Change Stoma Appliance in Older Rectal Cancer Patients with a Permanent Stoma

The effects of the continuing care bundle on self-efficacy, self-care knowledge, and the ability to change stoma appliances were tested, and as demonstrated in Table 2, no statistically significant differences were found between the two groups at discharge (both *P* > 0.05). However, the increased scores were displayed in the bundle group at 1-month and 3-months after discharge as compared with those in the control group (all *P* < 0.05). Higher levels of self-efficacy, self-care knowledge, and the ability to change stoma appliances were revealed after receiving the continuing care bundle (1-month and 3-months) than before (all *P* < 0.05).

### 3.3. The Effects of the Continuing Care Bundle on the Quality of Life of Older Rectal Cancer Patients with a Permanent Stoma

As shown in Table 3, there was no significant difference in any of the SF-36 subscales between the patients in the bundle group and control group at discharge (all *P* > 0.05). However, at one-month after discharge, the Bundle group had a higher score of GH and V than the control group (both *P* < 0.05). Moreover, at 3-month after discharge, except for BP and RE, the other SF-36 subscales, including PF, RP, GH, V, SF, and MH, were increased in patients given a continuing care bundle as compared to those with conventional care (all *P* < 0.05). There was no significant effect of conventional care on any of the SF-36 subscales at 1- and 3-months after discharge (all *P* > 0.05). In addition, as compared with the patients in the bundle group at discharge, those at 1- and 3-months after discharge showed higher levels of RP and V (all *P* < 0.05).

### 3.4. The Influence of the Continuing Care Bundle on Depression and Anxiety in Older Rectal Cancer Patients with a Permanent Stoma

As demonstrated in Table 4 and Figure 1, there was no statistically significant difference in the SDS scores between the Control and Bundle groups at discharge (*P*=0.781) nor was there a statistically significant difference in the SAS scores between these two groups (*P*=0.862). Furthermore, no significant differences were found in the SDS and SAS scores in Control groups at discharge and after discharge (all *P* > 0.05). However, alleviated depression and anxiety in older rectal cancer patients with a permanent stoma was found after given continuing care bundle, namely, the reduced SDS and SAS scores was revealed in Bundle groups at 1 and 3 months after discharge (all *P* < 0.05) with more patient showed mild depression and anxiety.

### 3.5. Comparison of Patient Satisfaction between the Two Groups

Based on the Likert 5-Point Scale measurement, the bundle group (completely dissatisfied: *n* = 5, dissatisfied: *n* = 14, partially satisfied: *n* = 13, satisfied: *n* = 8, and completely satisfied: *n* = 2) had higher patient satisfaction than the control group (completely dissatisfied: *n* = 2, dissatisfied: *n* = 5, partially satisfied: *n* = 12, satisfied: *n* = 16, and completely satisfied: *n* = 7, *χ*^2^ = 11.03, *P*=0.026, Figure 2).

## 4. Discussion

Although the stoma after rectal cancer surgery has obvious clinical benefits, it is well known that it also has various adverse effects on quality of life, cause major psychological handicap and physical stress, and impaired the patient's social health [10, 33]. Besides, the ensuing mortality rate of elderly patients in the first 6 months postoperation could be up to 57% in the first 6 months postoperation when anastomotic leakage occurs [6]. Therefore, appropriate care after discharge is necessary to improve the health outcomes for patients with stomas as it is rare for ostomates to stay at the hospital throughout the recovery process [27]. Evidence-based care related to postoperative care and rehabilitation of individuals with stomas after discharge can serve to improve continuity of care and to optimize patient care [34]. In this retrospective study, the patients in Bundle group received the continuing care bundle for 3 months, including the information-based (WeChat, telephone, etc.) hospital-family integration continuous care [22, 24], home visiting [25], and outpatient clinic management [26] and so on, which showed significantly improved self-care knowledge (the replacement period for stoma appliances, daily life precautions, and ostomy-related complications) as compared with those given conventional care with the enhanced ability to change stoma appliance.

Moreover, the HRQoL, which plays as an important role in understanding the patient's perspective was often impaired in patients with stoma [33]. We, therefore, assessed the HRQoL using the SF-36, an increasingly common in both research and clinical practice in patients with a stoma [35, 36]. The result revealed higher scores of GH and V in the bundle group at 1-month after discharge, as well as higher scores of PF, RP, GH, V, SF, and MH at 3-month after discharge than in the control group. Moreover, as compared with the patients in the bundle group at discharge, those at 1- and 3-months after discharge showed increased levels of RP and V. The studies mentioned above indicated that the continuing care bundle could improve the physical and mental component summary (PCS & MCS) in elderly patients with rectal cancer after radical resection with permanent stoma. Consistently, the evidence-based continuing care bundle was showed having an effective role in improving the quality of life in rectal cancer patients (age 56.98 ± 14.66 years) with temporary stomas [18].

A previous study also showed the stoma group reported higher levels of anxiety and depression than the nonstoma group [37]. As we know, the stoma patients have serious psychosocial problems owing to the insufficient psychological preparation for ostomy surgeries and the stoma-related complications [38, 39]. Moreover, using the combination of nursing intervention and early nutritional support could alleviate the psychological anxiety-depression of the patients who underwent preventive stoma reversion by evaluating SDS and SAS scores [40]. In the study, the attenuated depression and anxiety in older rectal cancer patients with a permanent stoma was found after given the continuing care bundle with the reduced SDS and SAS scores at 1 and 3 months after discharge, suggesting the continuing care bundle after discharge could effectively improve the adverse emotions of patients with a permanent stoma accompanied by increased patient satisfaction. However, this study has the following limitations: (1) Patients with a permanent stoma following rectal cancer resection were more likely to have more complications, which should be considered in further research using some sensitive indexes to assess the severity of stoma complications; (2) The results may not be generalised as the total number of study participants is not high, and repeated analysis is needed with a larger number of participants after the power calculation of sample size; (3) Another study to investigate the effect of continuing care bundle in elderly patients with rectal cancer after radical resection with temporary stoma would be performed in the future.

In conclusion, the continuing care bundle can serve as a comprehensive effectiveness intervention in elderly rectal cancer patients after radical resection with permanent stoma via increasing self-efficacy and self-care knowledge, enhancing the ability to change stoma appliances, reliving negative emotions, and improving quality of life, which also increases patient satisfaction.

## Figures and Tables

**Figure 1:** The number of patients in the control group (*n* = 42) and bundle group (*n* = 42) with the different degree of depression and anxiety. Note. Zung's self-rating depression scale (SDS) and self rating anxiety scale (SAS).

**Figure 2:** Comparison of the patient satisfaction between the control group (*n* = 42) and bundle group (*n* = 42).

**Table 1:** Demographic data and disease characteristics of the bundle group and control group.

Parameters	Control group (*n* = 42)	Bundle group (*n* = 42)	*P*
Age (years)	78.07 ± 8.02	76.02 ± 6.21	0.194
BMI	19.78 ± 1.72	20.13 ± 1.72	0.360
Gender			
Male	30	28	
Female	12	14	0.814
Educational level			
Lower level (≤9 years)	17	19	
Higher level (>9 years)	25	23	0.826
Medical payment method			
Self-paying	16	13	
Not self-paying	26	29	0.647
Living status			
Live alone	4	6	
Not live alone	38	36	0.738
Area of residence			
Urban	25	28	
Rural	17	14	0.652
Smoking status			
Current	9	11	
Former	23	25	
Never	10	6	0.526
TNM stage			
I	14	13	
II	21	25	
III	7	4	0.548
Grade differentiation			
Poor	10	12	
Moderate	12	15	
High	20	15	0.541
Preoperative adjuvant chemoradiotherapy			
Yes	15	17	
No	27	25	0.823
Postoperative adjuvant chemoradiotherapy			
Yes	28	24	
No	14	18	0.501

**Table 2:** The effects of the continuing care bundle on self-efficacy, self-care knowledge, and the ability to change stoma appliance.

	At discharge	1 month after discharge	3 months after discharge
*Self-efficacy*			
Control group (*n* = 42)	69.6 ± 15.24	72.43 ± 15.37	77.19 ± 16.77
Bundle group (*n* = 42)	70.79 ± 13.77	81.93 ± 14.78^*∗*^	93.33 ± 14.39^*∗*#^
*P*	0.7082	0.005	<0.001

*Self‐care knowledge*			
Control group (*n* = 42)	16.57 ± 4.53	17.53 ± 5.19	17.98 ± 5.24
Bundle group (*n* = 42)	17.29 ± 2.63	19.35 ± 3.86^*∗*^	21.86 ± 3.93^*∗*#^
*P*	0.379	0.025	<0.001

*Ability to change stoma appliance*			
Control group (*n* = 42)	18.95 ± 2.47	19.26 ± 3.89	19.74 ± 3.7
Bundle group (*n* = 42)	18.5 ± 3.29	23.19 ± 4.79^*∗*^	27.51 ± 5.09^*∗*#^
*P*	0.478	<0.001	<0.001

*Note*. ^*∗*^*P* < 0.05 and ^*#*^*P* < 0.05 indicated the significant difference as compared the patients at discharge and 3 months after discharge in bundle group, respectively.

**Table 3:** The effects of the continuing care bundle on the quality of life of older rectal cancer patients with a permanent stoma.

SF-36	At discharge			1-month after discharge			3-month after discharge		
	Control group (*n* = 42)	Bundle group (*n* = 42)	*P*	Control group (*n* = 42)	Bundle group (*n* = 42)	*P*	Control group (*n* = 42)	Bundle group (*n* = 42)	*P*
Global health (GH)	63.38 ± 20.16	66.00 ± 13.96	0.491	64.95 ± 19.86	72.40 ± 12.63	**0.043**	65.45 ± 19.07	76.40 ± 12.45^*∗*^	**0.003**
Physical function (PF)	59.14 ± 20.49	58.74 ± 20.55	0.928	60.07 ± 21.12	63.81 ± 20.66	0.415	61.38 ± 21.15	70.45 ± 17.25^*∗*^	**0.034**
Role physical (RP)	55.45 ± 10.05	54.67 ± 12.13	0.747	56.90 ± 9.55	60.64 ± 12.43^*∗*^	0.126	58.83 ± 9.72	67.14 ± 12.62^*∗*#^	**0.001**
Bodily pain (BP)	76.19 ± 11.50	76.48 ± 10.14	0.904	78.45 ± 10.28	77.57 ± 9.00	0.677	78.21 ± 8.45	78.52 ± 7.87	0.863
Vitality (V)	53.93 ± 24.99	52.95 ± 24.18	0.856	53.9 ± 25.58	67.67 ± 20.26^*∗*^	**0.009**	52.86 ± 25.18	71.05 ± 16.61^*∗*^	**0.001**
Social function (SF)	76.64 ± 21.21	75.07 ± 19.22	0.723	76.07 ± 21.5	79.74 ± 15.37	0.371	75.93 ± 21.13	84.33 ± 11.76^*∗*^	**0.027**
Role emotional (RE)	77.62 ± 11.78	76.76 ± 11.09	0.732	77.9 ± 11.96	76.29 ± 12.43	0.545	76.98 ± 12.82	76.74 ± 11.89	0.930
Mental health (MH)	68.67 ± 10.36	70.24 ± 11.15	0.505	68.43 ± 10.81	72.69 ± 11.2	0.080	69.12 ± 11.05	75.6 ± 11.18	**0.009**

*Note*. ^*∗*^*P* < 0.05 and ^*#*^*P* < 0.05 indicated the significant difference as compared the patients at discharge and 3 months after discharge in bundle group, respectively.

**Table 4:** The influence of the continuing care bundle on the depression and anxiety in older rectal cancer patients with a permanent stoma.

Time	SDS			SAS		
	Control group (*n* = 42)	Bundle group (*n* = 42)	*P*	Control group (*n* = 42)	Bundle group (*n* = 42)	*P*
At discharge	71.33 ± 14.96	72.17 ± 12.24	0.781	75.14 ± 11.46	74.67 ± 13.42	0.862
1 month after discharge	72.71 ± 13.36	65.93 ± 14.60	0.029	71.69 ± 14.47	62.40 ± 14.96^*∗*^	0.005
3 months after discharge	72.19 ± 11.49	55.71 ± 18.89^*∗*#^	<0.001	74.17 ± 12.43	52.55 ± 17.68^*∗*#^	<0.001

*Note*. Zung's self-rating depression scale (SDS) and self rating anxiety scale (SAS); ^*∗*^*P* < 0.05 and ^*#*^*P* < 0.05 indicated the significant difference as compared the patients in bundle group at discharge and 3 months after discharge, respectively.

## Data Availability

The data used to support the findings of this study are included within the article.
